The article "Occupational Disease and Injury in Malaysia: A Thematic Review of Literature from 2016 to 2021" was published in 2023. Journal: J Environ Public Health.

# Occupational Disease and Injury in Malaysia: A Thematic Review of Literature from 2016 to 2021

**DOI:** 10.1155/2023/1798434

**Published:** 2023-01-31

**Authors:** S. Maria Awaluddin, Maznieda Mahjom, Kuang Kuay Lim, Noor Syaqilah Shawaluddin, Tuan Mohd Amin Tuan Lah

**Affiliations:** Institute for Public Health, National Institutes of Health, Ministry of Health Malaysia, 40170 Bandar Setia Alam, Selangor, Malaysia

## Abstract

**Introduction:**

Working people are exposed to occupational hazards and are at risk of having occupational disease or injury in a rapidly industrializing country like Malaysia. This study aims to review and summarize the occupational disease and injury in Malaysia from 2016 to 2021.

**Methods:**

This study used PubMed and Scopus databases to conduct a systematic literature search using a set of keywords. The selected records dated from 1 January 2016 to 8 September 2021 were extracted into the Mendeley Desktop and ATLAS.ti 8 software. Systematic screening was conducted by two independent researchers and finalized by the third researcher. Data were coded and grouped according to the themes. The results were presented as the table for descriptive analysis and cross-tabulation between the themes.

**Results:**

A total of 120 records were included in this study. Under the theme of main health problems, the findings showed that mental health, infectious disease, and work-related musculoskeletal disorders are the top three problems being discussed in the literature for the working people in Malaysia. The findings also showed an increasing trend of mental health problems during pandemic COVID-19 years. In addition, hospital was the highest workplace where the occupational health problems were reported.*Discussion/Conclusion*. There was substantial work on the mental health problem, infectious diseases, and work-related musculoskeletal disorders as the main health problem among workers in Malaysia in the past five years. The employers must report any occupational health and injury case to the authority and prompt intervention can be initiated.

## 1. Introduction

People are exposed to occupational hazards or risks at the workplace which predisposes them to work-related injury or disease [1, 2]. In 2016, almost two million deaths were attributable to occupational risks and accounted for an estimated 2.1% of all deaths and 2.7% of the disease burden worldwide [3]. There are nineteen identified occupational risk factors with the most common factor being exposure to chemical hazards. The newly added occupational risk factor is exposure to long working hours (defined as working ≥55 hours per week) which pairs with the specific health outcomes of ischemic heart disease and stroke [4]. The occupational risks contribute to the total burden of chronic diseases such as 37% of all cases of back pain, 16% of hearing loss, 13% of chronic obstructive pulmonary disease, 11% of asthma, 8% of injuries, 9% of lung cancer, 2% of leukaemia, and 8% of depression [5].

Occupational disease or injury which occurs directly due to the nature of work and workplace environment may reduce workers' productivity, increase sick leave, and reduce the quality of life [6]. Substantial studies reported the prevalence of occupational disease and work-related disease in their country according to certain types of diseases such as asthma and work-related musculoskeletal disorders (WRMSDs) [7, 8]. Healthcare workers (HCWs) are the group who may exposed with biological hazards at the workplace as mention in previous studies [9, 10]. The International Labour Organisation (ILO) is responsible to compile the list of occupational diseases and classifying them into the disease caused by an agent (chemical, physical, biological) and the diseases according to the target organ (respiratory, skin, musculoskeletal, mental, and behavioural, occupational cancer and other diseases) [11, 12]. A similar classification is being used by the Department of Occupational Safety and Health Malaysia (DOSH) for surveillance data in Malaysia as well as in other countries [13]. Unfortunately, underreporting of occupational disease and injury is a known challenge for the stakeholders in estimating the true burden, worldwide. Taking China as the country with the largest working population of 776 million in 2018, more than 200 million of its workers are exposed to multiple risks including dust, chemicals, and poison, and this number is still underreported [14].

The DOSH published a yearly report on occupational poisoning and disease in Malaysia which shows increasing trends from 454 cases in 2005 to 9860 cases in 2019 [15]. The documentation of occupational disease is important for workers' compensation due to occupational disease or injury. Besides that, the information is useful for the stakeholders in planning for a preventive program at the national level in line with the healthy workplace campaign [5]. In Malaysia, the highest number of reported cases was recorded in the manufacturing sector and the highest number of diseases was the occupational noise-related hearing disorders [15].

Various studies were conducted concerning the occupational health issues in Malaysia in terms of occupational diseases and specific jobs [16–22], but the summarized literature was not found. Scarce evidence in the literature can summarize the recent occupational disease and injuries in Malaysia, and thus the study aims to review and summarize the occupational diseases and injuries being discussed in Malaysia from 2016 to 2021. Therefore, the underpinning of this paper is to review the occupational disease and work-related issues that have been discussed from the year 2016 to 2021.

## 2. Materials and Methods

A thematic review uses the basic concept of any systematic literature search by constructing a set of keywords for the initial record search in the established database. The term thematic review was introduced by Clarke and Braun as a process of identifying the important information, assigning a code to see the pattern, and summarizing the final themes [23]. The review process is facilitated by computer software, namely, ATLAS.ti, which was introduced by Dr. Zairul [24].

### 2.1. Search Strategy

In thematic review, the minimum number of databases required is at least two of the most common databases such as PubMed and Scopus [25]. The final search was conducted on 8 September 2021. The works of literature were searched for the period 1 January 2016 to 8 September 2021. A set of keywords was identified, and the search strings are shown in Table 1.

### 2.2. Inclusion and Exclusion Criteria

The summarized inclusion and exclusion criteria are shown in Figure 1.

Inclusion criteria:
  - Primary research on worked-related disease or injury
  - Conducted in Malaysia
  - Focused on standard working age of 15–64 years
  - Recent 5 years (1 January 2016–8 September 2021)
  - Cross-sectional, case-control studies or cohort
  - Mentioned prevalence, proportion of occupational disease, or injury
Exclusion criteria:
  - Any review articles
  - Focused on occupational hazard, intervention, or risk assessment without mentioning occupational disease or injury
  - Articles are written in languages other than English
  - Articles on review case based on DOSH report

### 2.3. Screening and Study Selection

The initial metadata of the two databases were exported to Mendeley Desktop for checking a duplicate record. A total of 164 articles were selected for review. Two researchers were assigned to screen the title, abstract, and full-text article, and any disagreement was resolved by the third researcher. Figure 1 shows the details of the screening process. The quality of study was assessed according to the National Heart Lung and Blood Institute guideline for observational cohort and cross-sectional studies [26].

### 2.4. Data Analysis

All the full-text articles were read by the researchers thoroughly to familiarize themselves with the data. The next step was to assign codes to the important text data followed by searching for themes, reviewing themes, and finally defining and naming the themes as described by Braun and Clarke [27]. A figure of word cloud was generated using ATLAS.ti 8. The descriptive analysis is conducted using Microsoft Excel and Atlas.ti.8 according to themes such as years of publication, main hazard, main health problems, working sector, workplace, occupation, main job title, and industry classification. The main job title was categorized according to the Malaysia Standard Classification of Occupations (MASCO) 2013 while Malaysia Standard Industrial Classification (MSIC) 2008 was used to classify the industry in Malaysia [28, 29].

## 3. Results

A descriptive analysis was conducted for a total of 120 articles. The quantitative findings are tabulated in Tables 2–4. The majority (65.5%) of the articles were produced by authors from medicine and health, engineering (13.3%), and biomedical (12.5%) fields as shown in Table 2. Approximately, 90.8% of the literature was based on a cross-sectional study design and 65.8% stated the sample of the respondent of more than 150 respondents. Word cloud was generated as shown in Figure 2 and shows the word musculoskeletal as the largest size equivalent to the number of literature.

There were seven sub-themes identified under the theme of main health problems as shown in Table 3. Table 3 also describes other themes such as type of hazards, main job title classification, industry classification, and the specific occupations' name according to the frequency and percentage.  Table 4 shows the cross-tabulation of the main health problem theme with the explanatory themes according to the number of articles. Each of the main health problem theme is explained further in the following qualitative section of in terms of the prevalence of specific health problem.

### 3.1. Qualitative Section

This section describes the seven main health problems in terms of the findings extracted from this review. All of the findings are summarized in Table 5.

#### 3.1.1. Mental Health Problems

A total of 29 articles discussed mental health problems among workers in Malaysia. Depression, anxiety and stress, emotional exhaustion, burnout, and workplace bullying were involved mainly among HCWs (15/29), while another half of the literature was spared for other occupations such as teachers (3/29) and office and general workers. A study conducted among railway workers found that the mean perceived stress was 18.8 which was above the 14/15 of the normal stress level [30]. Among teachers, the prevalence of depressive, anxiety, and stress symptoms was 43.0%, 68.0%, and 32.3%, respectively [31]. Studies conducted among shift workers in the manufacturing industry reported the problem of sleepiness [32, 33]. In terms of workplace bullying, 39.1% of participants reported ever being bullied in a study conducted by an insurance company among 5000 employees in Malaysia [34]. Workplace bullying was also investigated among HCW and the prevalence was 11.2% in one university hospital [35]. A study focusing on the mental health among intern doctors reported that depression, anxiety, and stress were 26.2%, 39.9%, and 29.7%, respectively, in a multi-hospital but a higher prevalence was noted in a study conducted in a single hospital [36, 37]. A study conducted by Abd Ghaffar et al. found that female gender and having depression were associated with lower quality of life among intern doctors [38]. The prevalence of burnout among all HCWs regardless of their specific occupation varies from 15.9% to 17.5% [39, 40] before the pandemic era, while a study conducted during the pandemic era showed that more than half of surveyed respondents reported burnout [41]. The contributing factors were higher works demands and fear of frequent exposure to COVID-19 patients [41, 42].

#### 3.1.2. Infectious Diseases

Infectious diseases among workers are best described according to the workplace environment or those who had contact with the biological hazard. Most of the literature provided the laboratory confirmation test of each biological hazard in their studies. The commonest occupational infectious disease in Malaysia is leptospirosis which can occur in animal farms, forests, palm oil plantations, wet markets, and municipal areas [43–49]. Many other infectious diseases are related to migrant workers who were detected having hydatid disease, blastocysts, entamoeba infections, *Giardia duodenalis*, worm infestations, and Toxoplasma infection. The prevalence of hydatid disease was 13.6% and 55.3% for leishmaniasis among the migrant worker respondents [50, 51]. A case of malaria was reported in Sabah from an immigrant rubber taper which caused the falciparum malaria outbreak in 2012 [52]. Besides that, migrant food handlers were reported as carriers of non-typhoidal Salmonella and practice poor hygiene practices that may cause food contamination by the pathogens [53, 54].

The recent literature discussing the COVID-19 pandemic put the HCWs at risk of COVID-19 infection. At the beginning of the pandemic, the rate of infections among HCWs was relatively low, except in a study conducted in Hospital Teluk Intan which caused the temporary closure of a few departments [55].

#### 3.1.3. Work-Related Musculoskeletal Disorders (WRMSDs)

WRMSDs may cause problems among the workers who need to use physical strength during working or in the sedentary group. It can be the hand-arm vibration syndrome and pain in a specific body part such as the neck, back, shoulder, and knee or any other body part which can be grouped as a musculoskeletal disorder. Studies conducted among hand-held grass-cutting workers and tyre shop workers highlighted the hand-arm vibration syndrome [21, 56, 57]. In terms of pain to the specific body part, low back pain was among the common problems and various studies reported the prevalence among HCWs: nurses (73.1%–76.5%), ambulance drivers (65.0%), and intern doctors (19.8%) [58–61]. Studies among dentists and dental auxiliaries reported upper back pain which involved the neck region [62, 63].

Various studies were conducted among teachers and noted the similar problems of WRMSD involving the lower back, neck, and shoulder [17, 64–66]. Besides HCWs and teachers, a study among commercial vehicle drivers also reported the prevalence of low back pain at 66.4% [67]. Those who worked in a factory were exposed to MSD due to ergonomic factors such as repetitive activities [68–70].

#### 3.1.4. Occupational Injury

The literature mainly focuses on non-fatal occupational injury than fatal injury. HCWs were at risk of needle stick injury and exposing them to the blood-borne disease [71–73]. Heat injury was described among outdoor workers such as farmers, forestry workers, and municipal workers [74–76]. Musculoskeletal injuries may happen among athletes, palm oil plantation workers, and construction workers ranging from muscle strains, sprains, and tears to falls from heights [16, 77, 78].

#### 3.1.5. Respiratory Problems

The respiratory problem among workers might include the problem of inhaling chemical hazards such as metal dust, endotoxin, pesticide, and any air pollutants. In terms of occupation, traffic police, firefighters, and farmers are among the at-risk workers for outdoor areas [79–81]. In contrast, indoor workers are also at risk of respiratory problems due to indoor dust. HCWs who worked in an orthopedic clinic might be exposed to dust from the plaster of Paris material [82]. Besides that, those who worked in mechanically ventilated offices in a tropical country were exposed to endotoxin from office dust [83]. Welders and factory workers should practice proper protection to prevent respiratory problems [84, 85].

#### 3.1.6. Cardiovascular Disease Risks

The trend of CVD risk prevalence is increasing in the general population and affecting the most productive population at an early age. The sedentary administrative workers were reported to have a prevalence of smoking, physical inactivity, and unhealthy diet which were at 20%, 50%, and 87%, respectively [86]. HCWs and firefighters were reported to have obesity problems despite their knowledge and nature of work [87–89]. A study conducted among secondary school teachers found that normal-weight participants had metabolic syndrome which put them at risk of progressing to CVD at a later age [90].

#### 3.1.7. Hearing Problems

Hearing loss is not uncommon among factory workers and in all workplaces which are exposed to the level of noise ≥85 dB. Two studies highlighted the hearing loss issue among factory workers while one study examined the noise level in the work area [91–93]. The prevalence of hearing loss was 73% among 146 respondents who worked in small and medium industries in Selangor [92]. Among the factors associated with hearing problems were occupational daily noise, length of service, infrequent use of HPD, age, male gender, and smoking status [91, 92].

## 4. Discussion and Areas for Further Research

This thematic review summarized the recent five years of literature discussing occupational disease and injury in Malaysia. Technically, DOSH under the Ministry of Human Resources is responsible to ensure the safety, health, and welfare of people at work. The department also produces the yearly statistic on occupational poisoning and diseases according to ten sectors under the 1994 Act. DOSH classified the ten sectors of work activities such as (1) manufacturing, (2) mining and quarrying, (3) construction, (4) hotels and restaurant, (5) agriculture, forestry and fishing, (6) transport, storage, and communication, (7) public services and statutory authorities, (8) utilities—gas, electricity, water, and sanitary services, (9) finance, insurance, real estate, and business services, and finally (10) wholesale and retail trades [15]. The Ministry of Human Resources adapts the International Standard Classification of Occupations (ISCO) to come out with Malaysian version of occupational classification, namely, MASCO, which can be accessed in public domain [29]. This study used the main job title classification to describe the specific occupation name.

Besides Ministry of Human Resources, the Department of Statistics Malaysia (DOSM) conducts the Labour Force Survey to highlight the employment and unemployment rates. The labour force survey used the updated version of MSIC in 2008 consisting of the updated version of industry classification with the current 20 groups of industries from the only nine groups for the year before 2000. The report also stated that the highest number of workers were in Group C (manufacturing) followed by Group G (wholesale and retail trade; repair of motor vehicles and motorcycles), Group I (accommodation and food service activities), Group A (agriculture, forestry, and fishing), and Group F (construction) [94]. DOSM as the main function of recording the general population statistic differs in the industry classification from DOSH because DOSM needs to update the classification according to the recent industrial development. A standard classification should be used by the authority bodies in order to minimize the overlapping job scope and underreporting issues among working people [13].

This thematic review found that a higher number of literature focused on Group Q (human health and social work activities) followed by Group A, Group C, Group O (public administration and defense; compulsory social security), and Group P (education) [15]. The possible reason for these findings is due to the recent pandemic (COVID-19) which affected the HCW group in terms of psychosocial, ergonomic, and biological hazards. Those who work in manufacturing industries might be exposed to the physical hazard while those in agriculture may have zoonosis infection [93, 95]. The increasing number of non-communicable diseases such as diabetes, hypertension, metabolic syndrome, and obesity might affect those who were in sedentary work style [86].

Traditionally, any occupational diseases were reported to DOSH as the main authority for further investigation. The highest reported health problem to the DOSH was occupational noise-related hearing loss, but this theme was less discussed recently. The literature discussed more biological hazards referring to COVID-19 which affected the healthcare workers. The occupational disease highlighted in the literature may not be reported to the DOSH because it is mainly for educational purposes. The DOSH reported of five, zero, four, and one confirmed cases of workers who had a psychosocial problem in 2017, 2018, 2019, and 2020, respectively, which contradicted the abundant literature on mental health as found in this study. One of the challenges reported by the previous study is the underreporting problem of the occupational disease cases which affects the worldwide surveillance system [13]. The current trend showed that occupational diseases reported to DOSH traditionally are focusing on workers in manufacturing and construction industries while those in other industries such as education and public administration may be left behind. With the current situation of the post-pandemic era, a higher number of mental health problems arise but may not be reported to the authority. Thus, collaborative work among the authorities is needed to increase reporting of any cases suspected of psychosocial problems.

The recent work of WHO and ILO found that the risk of long working hours defined as ≥55 hours/week is paired with the health outcomes of ischemic disease and stroke [96]. The situation during the pandemic which exposed a group of frontliners including the HCWs and public administration and defense staff to the long working hours may contribute to a sudden cardiovascular attack. However, this may need more work since CVD is multi-factorial which includes individual lifestyle, family history, sedentary working type, and mental health problems. Even before the pandemic era, a younger age patient was seen for having a sudden attack of myocardial infarction which led to a new recommendation of CVS screening as early as 30 years [97].

According to the Occupational Safety and Health Master Plan 2021–2025 (OSHMP25), one of the indicators aims to increase the occupational diseases/injuries reported by 30% in 2025 [15]. This may need collaborative work among employers in both public and private industries to be responsible for data reporting. Besides that, the small and medium industries lack in providing the proper channel of healthcare service where the workers' health assessments are not conducted by the occupational health doctors but are treated as normal patients in the local health facility [98]. The challenges are faced by primary care doctors who may be less trained in occupational health [98].

### 4.1. Strengths and Limitations of the Study

This study used a thematic review concept to give an overview of the recent issues related to occupational disease and injury in Malaysia. The number of reviewed articles was more than hundreds of articles, and it was managed using the Mendeley reference manager and ATLAS.ti 8 for the qualitative data analysis. The majority of the selected studies are cross-sectional study designs, and nearly three-quarters had adequate sample sizes. Even though the cross-sectional study design lacks a causal relationship, the important content such as the type of main health problems and their prevalence can be extracted from the selected studies. This generated study's findings via thematic and content analysis managed to answer the research question.

## 5. Conclusion

This study summarized the literature on the evidence of occupational diseases in Malaysia over the recent five years. The substantial number of literature on mental health problems may not be in line with the reported cases in DOSH. A psychosocial factor may be the main hazard for workers in Malaysia, worsening with the pandemic (COVID-19). This study highlighted that there are discrepancies between issues being discussed in literature among workers with occupational diseases or injuries being reported to the relevant authority. Therefore, working people in Malaysia should be advised to seek help if they are facing any occupational hazards at the workplace. Collaborative work between agencies must be strengthened towards providing a better healthcare service for working people.

## Figures and Tables

**Figure 1:** Inclusion and exclusion criteria in the thematic review.

**Figure 2:** Word cloud of the recent occupational health issues in Malaysia.

**Table 1:** Search strings from Scopus and PubMed.

Databases	Search string	Initial result
Scopus	TITLE-ABS-KEY ((occupation^*∗*^ OR job OR work^*∗*^ OR career OR profession OR employee^*∗*^ OR work-related OR worksite OR workplace) AND (disease^*∗*^ OR injury^*∗*^ OR problem^*∗*^ OR accident^*∗*^ OR illness^*∗*^) AND (Malaysia))	1519
	Filter 5 year	

PubMed	(occupation^*∗*^ OR job OR work^*∗*^ OR career OR profession OR employee^*∗*^ OR work-related OR worksite OR workplace) AND (disease^*∗*^ OR injury^*∗*^ OR problem^*∗*^ OR accident^*∗*^ OR illness^*∗*^) AND Malaysia	1752
	(“occupation^*∗*^”[All Fields] OR “job”[All Fields] OR “work^*∗*^”[All Fields] OR (“career”[All Fields] OR “careers”[All Fields]) OR (“occupations”[MeSH Terms] OR “occupations”[All Fields] OR “profession”[All Fields] OR “professions”[All Fields] OR “profess”[All Fields] OR “professed”[All Fields] OR “professing”[All Fields] OR “profession s”[All Fields]) OR “employee^*∗*^”[All Fields] OR “work-related”[All Fields] OR (“workplace”[MeSH Terms] OR “workplace”[All Fields] OR “worksite”[All Fields] OR “worksites”[All Fields]) OR (“workplace”[MeSH Terms] OR “workplace”[All Fields] OR “workplaces”[All Fields] OR “workplace s”[All Fields])) AND (“disease^*∗*^”[All Fields] OR “injury^*∗*^”[All Fields] OR “problem^*∗*^”[All Fields] OR “accident^*∗*^”[All Fields] OR “illness^*∗*^”[All Fields]) AND (“Malaysia”[MeSH Terms] OR “Malaysia”[All Fields] OR “Malaysia s”[All Fields])	
	Translations career: “career”[All Fields] OR “careers”[All Fields]	
	Profession: “occupations”[MeSH Terms] OR “occupations”[All Fields] OR “profession”[All Fields] OR “professions”[All Fields] OR “profess”[All Fields] OR “professed”[All Fields] OR “professing”[All Fields] OR “profession's”[All Fields]	
	Worksite: “workplace”[MeSH Terms] OR “workplace”[All Fields] OR “worksite”[All Fields] OR “worksites”[All Fields]	
	Workplace: “workplace”[MeSH Terms] OR “workplace”[All Fields] OR “workplaces”[All Fields] OR “workplace's”[All Fields]	
	Malaysia: “Malaysia”[MeSH Terms] OR “Malaysia”[All Fields] OR “Malaysia's”[All Fields]	
	Filter 5 year	

**Table 2:** Descriptive analysis of the literature on occupational disease and injury (2016–2021).

Descriptive themes	*N* = 120	%
Authors' department		
Medicine and health	78	65.0
Engineering	16	13.3
Biomedical	15	12.5
Science and technology	3	2.5
Dentistry	2	1.7
Environment	2	1.7
Veterinary	2	1.7
Economic	1	0.8
Education	1	0.8
Occupational health issue		
Occupational disease	106	88.3
Occupational injury	14	11.7
Sample size of the study		
150 and above	79	65.8
Below 150	39	32.5
Not mentioned	2	1.7
Study design		
Cross-sectional	109	90.8
Case-control	8	6.7
Others	3	2.5
Working sector		
Public	52	43.3
Private	68	56.7
Nationality of the worker		
Malaysian	102	85.0
Non-Malaysian	18	15.0

**Table 3:** The thematic content analysis of the literature on occupational disease and injury (2016–2021).

Themes	*n*	%
Main hazard		
Physical	42	35.0
Biology	30	25.0
Psychosocial	29	24.2
Chemical	14	11.7
Others	5	4.2
Main health problem		
Mental health (MH)	29	24.2
Infectious disease (infection)	28	23.3
WRMSDs	28	23.3
Injury	14	11.7
Respiratory problems (R)	12	10.0
Cardiovascular disease risks (CVDs)	6	5.0
Hearing problems (HPs)	3	2.5
Main job title classification (MASCO 2020)		
Group 1: managers and senior officials	1	0.8
Group 2: professionals	21	17.5
Group 3: associate professional and technical officers	4	3.3
Group 4: administration and secretarial occupations	5	4.2
Group 5: personal service occupations	9	7.5
Group 6: skilled agricultural, forestry, livestock, and fishery workers	15	12.5
Group 7: craft and related trade workers	4	3.3
Group 8: plant and machine operators and assemblers	15	12.5
Group 9: elementary occupations	20	16.7
Group 0: armed forces	2	1.7
Not specified: more than one groups	24	20.0
Specific occupation's name and its MASCO group		
^*∗*^Healthcare worker	32	26.7
Group 8: factory worker	14	11.7
Group 8: palm oil plantation worker	11	9.2
Group 2: teacher	8	6.7
Group 6: farmer	7	5.8
Group 9: general worker	6	5.0
^*∗*^Office worker	6	5.0
Group 3: university staff	4	3.3
Group 5: firefighters and traffic police	4	3.3
Group 6: animal slaughter	2	1.7
Group 0: army recruit	2	1.7
Group 2: athlete	2	1.7
^*∗*^Employee	2	1.7
Group 5: food handler	2	1.7
Group 9: hand-held grass-cutting worker	2	1.7
Group 7: welder	2	1.7
Group 6: wet market worker	2	1.7
Group 7: commercial vehicle driver	1	0.8
Group 9: construction worker	1	0.8
Group 1: contractor	1	0.8
Group 6: dog handler	1	0.8
Group 9: domestic waste collector	1	0.8
Group 9: forestry worker	1	0.8
Group 9: landscape worker	1	0.8
^*∗*^Railway worker	1	0.8
Group 6: rubber tapper	1	0.8
Group 8: sex worker	1	0.8
Group 6: tea plucker	1	0.8
Group 6: tyre shop worker	1	0.8
Industry classification (MSIC 2008)		
Q: human health and social work activities	32	26.7
A: agriculture, forestry, and fishing	18	15.0
C: manufacturing	17	14.2
O: public administration and defense; compulsory social security	12	10.0
P: education	11	9.2
E: water supply; sewerage, waste management, and remediation activities	6	5.0
I: accommodation and food service activities	4	3.3
R: arts, entertainment, and recreation	3	2.5
F: construction	2	1.7
H: transportation and storage	2	1.7
G: wholesale and retail trade; repair of motor vehicles and motorcycles	1	0.8
Not specified: more than one industry	12	10.0
Specific workplace		
Hospital	28	23.3
Factory	16	13.3
Farm	15	12.5
Not specified	9	7.5
School	8	6.7
Office	6	5.0
Higher education	5	4.2
Palm oil plantation	5	4.2
Road	5	4.2
Municipal	4	3.3
Clinic	3	2.5
Forest	3	2.5
Abattoir	2	1.7
Food stall	2	1.7
Site work	2	1.7
Sport centre	2	1.7
Wet market	2	1.7
Animal shelter	1	0.8
Tea plantation	1	0.8
Tyre shop	1	0.8

^*∗*^No specific group of MASCO can be coded; it involves many groups.

**Table 4:** Cross-tabulation of the main health problem theme with the explanatory themes according to the number of articles.

Explanatory themes	Main health problems						
	MH	Infection	WRMSDs	Injury	R	CVDs	HPs
Year of publication							
2016	1	5	2	2	2	3	2
2017	2	7	6	2	1	1	1
2018	2	5	6	1	2	—	—
2019	6	3	5	4	3	—	—
2020	9	4	7	2	4	2	—
2021	9	4	2	3	—	—	—
Main hazard							
Physical	—	—	28	11	—	—	3
Biology	—	28	—	2	—	—	—
Psychosocial	29	—	—	—	—	—	—
Chemical	—	—	—	1	12	1	—
Ergonomic	—	—	—	—	—	5	—
Nationality of the worker							
Malaysian	27	17	26	11	12	6	3
Non-Malaysian	2	11	2	3	—	—	—
Working sector							
Public	20	3	15	3	5	6	—
Private	9	25	13	11	7	—	3
Workplace							
Abattoir	—	1	—	1	—	—	—
Animal shelter	—	1	—	—	—	—	—
Clinic	—	1	1	—	—	1	—
Factory	3	—	4	1	5	—	3
Farm	—	13	—	1	1	—	—
Food stall	—	2	—	—	—	—	—
Forest	—	1	1	1	—	—	—
Higher education	1	—	4	—	—	—	—
Hospital	15	3	5	3	1	1	—
Municipal	—	1	1	1	1	—	—
Office	1	—	2	—	1	2	—
Palm oil plantation	—	2	—	3	—	—	—
Road	—	—	2	—	3	—	—
School	3	—	4	—	—	1	—
Site	—	—	—	1	—	1	—
Sport centre	—	—	—	2	—	—	—
Tea plantation	—	—	1	—	—	—	—
Tyre shop	—	—	1	—	—	—	—
Wet market	—	2	—	—	—	—	—
Occupation							
Construction worker	—	—	—	1	—	—	—
Firefighter and policeman	—	—	—	—	3	1	—
Tea plucker	—	—	1	—	—	—	—
Tyre shop	—	—	1	—	—	—	—
Wet market worker	—	2	—	—	—	—	—
Animal slaughter	—	1	—	1	—	—	—
Army recruit	—	1	1	—	—	—	—
Athletes	—	—	—	2	—	—	—
Commercial vehicle driver	—	—	1	—	—	—	—
Dog handler	—	1	—	—	—	—	—
Domestic waste collector	—	—	—	—	1	—	—
Employee (not specified)	2	—	—	—	—	—	—
Factory worker	3	—	3	1	4	—	3
Farmer	—	5	—	1	1	—	—
Food handler	—	2	—	—	—	—	—
Forestry worker	—	—	—	1	—	—	—
G7 class of contractor	1	—	—	—	—	—	—
General worker	2	2	1	1	—	—	—
Hand-held grass-cutting worker	—	—	2	—	—	—	—
Healthcare worker	15	4	6	3	1	3	—
Landscape worker	—	—	1	—	—	—	—
Office worker	1	—	3	—	1	1	—
Palm oil plantation worker	—	8	—	3	—	—	—
Railway worker	1	—	—	—	—	—	—
Rubber tapper	—	1	—	—	—	—	—
Sex worker	—	1	—	—	—	—	—
Teacher	3	—	4	—	—	1	—
University staff	1	—	3	—	—	—	—
Welder	—	—	1	—	1	—	—
Main job title classification (MASCO 2020)							
Group 1: managers and senior officials	1	—	—	—	—	—	—
Group 2: professionals	10	1	7	2	—	1	—
Group 3: associate professional and technical officers	—	—	4	—	—	—	—
Group 4: administration and secretarial occupations	—	—	3	—	1	1	—
Group 5: personal service occupations	—	2	1	—	3	2	—
Group 6: skilled agricultural, forestry, livestock, and fishery workers	—	10	1	3	1	—	—
Group 7: craft and related trade workers	—	1	4	—	—	—	—
Group 8: plant and machine operators and assemblers	2	1	2	3	4	—	3
Group 9: elementary occupations	3	9	4	3	1	—	—
Group 0: armed forces	—	1	1	—	—	—	—
Industry classification (MSIC 2008)							
A: agriculture, forestry, and fishing	—	10	1	6	1	—	—
C: manufacturing	3	—	5	1	5	—	3
E: water supply; sewerage, waste management, and remediation activities	—	1	3	1	1	—	—
F: construction	1	—	—	1	—	—	—
G: wholesale and retail trade; repair of motor vehicles and motorcycles	—	—	1	—	—	—	—
H: transportation and storage	1	—	1	—	—	—	—
I: accommodation and food service activities	—	4	—	—	—	—	—
O: public administration and defense; compulsory social security	1	1	4	—	4	2	—
P: education	4	—	6	—		1	—
Q: human health and social work activities	15	4	6	3	1	3	—
R: arts, entertainment and recreation	—	1	—	2	—	—	—

Mental health (MH), work-related musculoskeletal disorders (WRMSDs), respiratory problems (R), cardiovascular disease risks (CVDs), and hearing problems (HPs).

**Table 5:** Table of the literature included for manuscript entitled “the occupational disease and injury in Malaysia: a thematic review of literature from 2016 to 2021.”

ID	Author	Years	Measure	Main hazard	Main health problems	Workplace	Occupation	MASCO	MSIC	SS	SD	Findings
(1)	Othman and Sivasubramaniam	2019	Depression, anxiety, and stress	Psychosocial	Mental health	School	Teacher	Professionals	P	1	1	Prevalence of depression (43.0%), anxiety (68.0%), and stress (32.3%)
(2)	Hashim and Samad	2019	Psychological distress	Psychosocial	Mental health	School	Teacher	Professionals	P	1	1	Respiratory problems were the significant risk factors for poor mental health status (*p* < 0.001) of teachers in schools
(3)	Omar and Sallehudin	2018	Psychological distress	Psychosocial	Mental health	NS	Contractor	Managers and senior officials	F	2	1	Work demand is the main factor contributing to the high-pressure jobs
(4)	Rasdi et al.	2019	Psychological distress	Psychosocial	Mental health	Factory	Factory worker	Elementary occupations	C	1	1	36.6% of respondents reported to have job strain and 53.6% reported to have excessive daytime sleepiness
(5)	Noor and Shaker	2017	Psychological distress	Psychosocial	Mental health	NS	General worker	Elementary occupations	NS	2	2	Workplace discrimination was positively related to psychological distress
(6)	Chan et al.	2019	Workplace bullying	Psychosocial	Mental health	NS	Employee	NS	NS	1	1	A total of 2045 (39.1%) participants reported ever being bullied
(7)	Awai et al.	2021	Workplace bullying	Psychosocial	Mental health	Hospital	Healthcare worker	NS	Q	1	1	Prevalence of workplace bullying in this sample was 11.2%
(8)	Al-Dubai et al.	2016	Psychological distress	Psychosocial	Mental health	NS	Railway worker	NS	H	1	1	Mean (SD) perceived stress was 18.8 (4.3), with above 15 as the normal cutoff score
(9)	Zakaria et al.	2019	Burnout	Psychosocial	Mental health	Hospital	Healthcare worker	Professionals	Q	1	1	Among the burnout features were fatigue with 52.2% and frequent physical illness and feel unappreciated with 48.6% and 45.9%, respectively. The job-related issues which predisposed to burnout were demand coping with an angry public with 70.2%, job overload 63.9%, lack clear guideline or rapid program changes 54%, and pay too little 53.1%.
(10)	Woon and Tiong	2020	Burnout	Psychosocial	Mental health	Hospital	Healthcare worker	NS	Q	1	1	Burnout rates were 17.5% (personal burnout), 13.9% (work burnout), and 6.0% (client burnout)
(11)	Boo et al.	2018	Burnout	Psychosocial	Mental health	Hospital	Healthcare worker	Professionals	Q	1	1	15.9% of the respondents experienced high burnout syndrome
(12)	Khoo et al.	2017	Emotional exhaustion	Psychosocial	Mental health	Hospital	Healthcare worker	Professionals	Q	1	1	High and moderate emotional exhaustion was reported by 25.4% and 24.4% doctors, respectively
(13)	Ismail et al.	2021	Depression, anxiety, and stress	Psychosocial	Mental health	Hospital	Healthcare worker	Professionals	Q	1	1	Prevalence of stress, anxiety, and depression was 29.7%, 39.9%, and 26.2%
(14)	Abd Gaffar et al.	2021	Quality of life	Psychosocial	Mental health	Hospital	Healthcare worker	Professionals	Q	1	1	Being female and having depression were found to be associated with lower QOWL
(15)	Minn et al.	2019	Depression, anxiety, and stress	Psychosocial	Mental health	Hospital	Healthcare worker	Professionals	Q	1	1	Prevalence of psychiatric morbidities such as depression (42%), anxiety (50%), and stress (42.7%)
(16)	Ng et al.	2020	Depression, anxiety, and stress	Psychosocial	Mental health	Hospital	Healthcare worker	NS	Q	2	1	HCWs undergoing contact swabbing and quarantine are vulnerable to depression, anxiety, and stress
(17)	Mohd Fauzi et al.	2020	Fatigue	Psychosocial	Mental health	Hospital	Healthcare worker	Professionals	Q	1	1	Work demands generally worsen, while recovery experiences protect mental health during the COVID-19 pandemic with the caveat of the role of detachment experiences
(18)	Woon et al.	2020	Depression, anxiety, and stress	Psychosocial	Mental health	Hospital	Healthcare worker	NS	Q	1	1	Prevalence rates of depression, anxiety, and stress were 21.8%, 31.6%, and 29.1%, respectively
(19)	Noor et al.	2021	Anxiety	Psychosocial	Mental health	Hospital	Healthcare worker	NS	Q	1	2	Non-frontline healthcare providers require psychological support similar to that of frontline healthcare providers during the COVID-19 pandemic
(20)	Roslan et al.	2021	Burnout	Psychosocial	Mental health	Hospital	Healthcare worker	NS	Q	1	1	More than half of Malaysian healthcare workers in this sample experienced burnout
(21)	Sze Kiat et al.	2021	Depression, anxiety, and stress	Psychosocial	Mental health	Hospital	Healthcare worker	NS	Q	2	1	Healthcare workers had mild anxiety, with the majority experiencing mild stress (57.1%) and almost half of the respondents experiencing mild depression (41%)
(22)	Sahimi et al.	2021	Suicidal ideation	Psychosocial	Mental health	Hospital	Healthcare worker	NS	Q	1	1	Current suicidal ideation (19/171) and clinical depression (17/171) were good HRQOL with the mean score of overall HRQOL was 72.42 ± 14.99. 11.1 and 9.9%
(23)	Ashri et al.	2021	Quality of life	Psychosocial	Mental health	Office	Office worker	NS	O	1	1	Good HRQOL with the mean score of overall HRQOL was 72.42 ± 14.99.
(24)	Nazali et al.	2021	Quality of life	Psychosocial	Mental health	Higher education	University staff	NS	P	1	1	Participants had low QOL in the domains of physical health (P-QOL) (11.2%), psychological health (PSY-QOL) (9.7%), social relationships (SR-QOL) (19.1%), and environment (E-QOL) (14.4%)
(25)	Shahril Abu Hanifah and Ismail	2020	Fatigue	Psychosocial	Mental health	Factory	Factory worker	Plant and machine operators and assemblers	C	1	1	General fatigue (54.5%)
(26)	Htay et al.	2020	Psychological distress	Psychosocial	Mental health	NS	General worker	Elementary occupations	NS	1	1	79.2% had poor mental well-being according to the WHO-5 scale
(27)	Lee and Lai	2020	Depression, anxiety, and stress	Psychosocial	Mental health	School	Teacher	Professionals	P	1	1	Majority of the female teachers tend to have normal level for stress, anxiety, and depression
(28)	Ah et al.	2020	Sleepiness	Psychosocial	Mental health	Factory	Factory worker	Plant and machine operators and assemblers	C	1	1	Sleepiness among shift workers found to be increased by the end of the shift. Around 30% of workers did not have an adequate amount of daily sleep.
(29)	Jalali et al.	2020	Workplace bullying	Psychosocial	Mental health	NS	Employee	NS	NS	2	1	Workplace bullying has a positive impact on job insecurity as well as emotional exhaustion while also having a positive indirect effect on emotional exhaustion through job insecurity
(30)	Kisomi et al.	2016	Tick-borne diseases	Biology	Infection	Farm	Farmer	Skilled agricultural, forestry, livestock, and fishery workers	A	1	1	More than half of the farmworkers (*n* = 91) reported an experience of tick bites
(31)	Shamsul et al.	2016	*Escherichia coli*	Biology	Infection	Abattoir	Animal slaughter	Skilled agricultural, forestry, livestock, and fishery workers	A	1	1	Prevalence of 9.7% was recorded for all samples during work for *Escherichia coli* O157 : H7 isolated on the hands of before and after work. For non-O157 : H7, total prevalence of 33.3% during work and 13% after work was obtained.
(32)	Bamaiyi et al.	2017	Seroprevalence of brucellosis	Biology	Infection	Farm	Farmer	Skilled agricultural, forestry, livestock, and fishery workers	A	1	1	Seroprevalence of brucellosis among farmers and non-farmers (veterinary technical staff and others) of 446 people studied was 1.35% (95% CI = 0.28–2.42)
(33)	Najib et al.	2020	Fasciola infection	Biology	Infection	Farm	Farmer	Skilled agricultural, forestry, livestock, and fishery workers	A	2	1	Serological screening revealed 60 (67%) participants positive for anti-Fasciola IgG antibody
(34)	Khan et al.	2020	Hydatid disease	Biology	Infection	Farm	General worker	Elementary occupations	A	1	1	13.6% of the migrant workers were found to be seropositive for hydatid disease
(35)	Jeffree et al.	2018	Malaria	Biology	Infection	Farm	Rubber tapper	Skilled agricultural, forestry, livestock, and fishery workers	A	1	2	Malarial attack rate was 2.3%, 6/11 smears have gametocyte, and the case fatality rate was 9.1%
(36)	Kho et al.	2017	Rickettsia disease	Biology	Infection	Farm	Farmer	Skilled agricultural, forestry, livestock, and fishery workers	A	2	1	Indigenous community had significantly higher seropositivity rates for *R. conorii* (*p* < 0.001) and *R. felis* (*p* < 0.001), as compared to blood donors from urban (*n* = 61). Similarly, higher seropositivity rates for *R. conorii* (*p*=0.046) and *R. felis* (*p* < 0.001) were noted for animal farm workers, as compared to urban blood donors.
(37)	Lee et al.	2017	Bacterial infections	Biology	Infection	Food stall	Food handler	Personal service occupations	I	2	1	Moderate levels of food safety knowledge (61.7%) with good attitude (51.9/60) and self-reported practices (53.2/60). It is noteworthy that the good self-reported practices were not reflected in the microbiological assessment of food handlers' hands, in which 65% of the food handlers examined had a total aerobic count ≥20 CFU/cm^2^ and Salmonella was detected on 48% of the food handlers' hands.
(38)	Woh et al.	2017	Salmonella carriers	Biology	Infection	Food stall	Food handler	Personal service occupations	I	1	1	Nine (2.8%) stool samples were confirmed to be Salmonella positive
(39)	Wickersham et al.	2017	Sexual transmitted diseases	Biology	Infection	NS	Sex worker	Personal service occupations	R	1	1	Screening for STI was low. Inconsistent condom use and drug use during sex work were not uncommon.
(40)	Noor Azian et al.	2016	Leishmaniasis	Biology	Infection	Palm oil plantation	Palm oil plantation worker	Elementary occupations	NS	1	1	55.3% were seropositive, with the highest was among the Nepalese (68.6%), followed by Indians (62.2%), Bangladeshi (54.9%), Myanmar (44.4%), Vietnamese (25.8%), and Indonesian (25.6%)
(41)	Mohd Ridzuan et al.	2016	Leptospirosis	Biology	Infection	Palm oil plantation	Palm oil plantation worker	Plant and machine operators and assemblers	A	1	1	100 of 350 workers tested positive for leptospiral antibodies, hence a seroprevalence of 28.6% (95% CI 23.8% to 33.3%)
(42)	Rahman et al.	2018	Leptospirosis	Biology	Infection	Wet market	Wet market worker	Skilled agricultural, forestry, livestock, and fishery workers	I	1	1	Seroprevalence for leptospirosis among the respondents was 33.6% (95% CI = 27.5, 39.7)
(43)	Samsudin et al.	2018	Leptospirosis	Biology	Infection	Wet market	Wet market worker	Skilled agricultural, forestry, livestock, and fishery workers	I	1	1	Seroprevalence of leptospirosis among healthy workers was 46.3%
(44)	Goh et al.	2019	Leptospirosis	Biology	Infection	Animal shelter	Dog handler	Skilled agricultural, forestry, livestock, and fishery workers	A	1	1	A total of 22.2% of dogs and 21.7% of dog handlers were seropositive
(45)	Binti Daud et al.	2018	Leptospirosis	Biology	Infection	Farm	Farmer	Skilled agricultural, forestry, livestock, and fishery workers	A	2	1	Seroprevalence of leptospiral antibodies was 72.5% (95% CI 63.5% to 80.1%) and the prevalence of pathogenic *Leptospira* in the cattle farms environment was 12.1% (95% CI 8.4% to 17.0%)
(46)	Neela et al.	2019	Leptospirosis	Biology	Infection	Forest	Army recruit	Armed forces	O	2	1	Among 12 patients, two (2/12; 16.6%) were confirmed positive for leptospirosis by microscopic agglutination test (MAT with titres 400–800)
(47)	Atil et al.	2020	Leptospirosis	Biology	Infection	Municipal	General worker	Elementary occupations	E	1	1	Positive *Leptospira* was 9.4% (95% CI: 6.8–12.8). Urban sweepers and lorry drivers made up the highest proportion of positive *Leptospira* respondents, contributing 15.5% and 9.4%, respectively
(48)	Mani et al.	2021	COVID-19 infection	Biology	Infection	Clinic	Healthcare worker	Professionals	Q	1	1	Most dentists limited their clinical services during the MCO and resumed work once restrictions were lifted during the C-MCO and R-MCO. Many reported adopting appropriate precautionary measures to mitigate the spread of COVID-19.
(49)	Tan-Loh and Cheong	2021	COVID-19 infection	Biology	Infection	Hospital	Healthcare worker	NS	Q	2	1	47 HCWs in HTI tested positive for COVID-19. 7 patients (15.2%) had at least more than one comorbidity.
(50)	Wan et al.	2021	COVID-19 effect	Biology	Infection	Hospital	Healthcare worker	NS	Q	1	1	One-third (35.2%) were symptomatic, with sore throat (23.6%), cough (19.8%), and fever (5.0%) being the most commonly reported symptoms. A total of 17 healthcare workers tested positive for COVID-19, with a prevalence of 0.3% among all the healthcare workers. Risk category and presence of symptoms were associated with a positive COVID-19 test (*p* < 0.001). Fever (*p* < 0.001), cough (*p*=0.003), shortness of breath (*p*=0.015), and sore throat (*p*=0.002) were associated with case positivity.
(51)	Woon et al.	2021	COVID-19 infection	Biology	Infection	Hospital	Healthcare worker	NS	Q	1	1	One hundred and fifteen (29%) participants claimed to have had contact with known COVID-19 persons outside of their workplace
(52)	Sahimin et al.	2020	Blastocystis	Biology	Infection	Farm	Palm oil plantation worker	Elementary occupations	NS	1	1	A third of the study cohort (30.9%; *n* = 68/220) screened were infected with *Blastocystis* sp. predominantly with ST3 (54.5%; *n* = 12), followed by ST1 (36.4%; *n* = 8) and ST2 (9.1%; *n* = 2)
(53)	Sahimin et al.	2019	Entamoeba infections	Biology	Infection	Farm	Palm oil plantation worker	Elementary occupations	NS	1	1	Seroprevalence of 7.4% (*n* = 36; CL95 = 5.3–10.1%) with only one factor statistically associated with seropositivity of anti-amoebic antibodies, i.e., years of residence in Malaysia (*χ*^21^ = 4.007, *p*=0.045)
(54)	Sahimin et al.	2018	*Giardia duodenalis*	Biology	Infection	Farm	Palm oil plantation worker	Elementary occupations	NS	1	1	10.8% (*n* = 42) were found to be positive with *Giardia* spp. and 3.1% (*n* = 12) were found to be positive with *Cryptosporidium* spp. infections
(55)	Sahimin et al.	2017	Hookworm	Biology	Infection	Farm	Palm oil plantation worker	Elementary occupations	NS	1	1	51 samples (13.1%) were positive by microscopy for hookworm infections
(56)	Sahimin et al.	2017	Toxoplasma gondii infection	Biology	Infection	Farm	Palm oil plantation worker	Elementary occupations	NS	1	1	Seroprevalence of *T. gondii* was 57.4% (*n* = 278; 95% CI: 52.7–61.8%)
(57)	Sahimin et al.	2016	Intestinal parasitic infections	Biology	Infection	Farm	Palm oil plantation worker	Elementary occupations	NS	1	1	Prevalence of infections with *A. lumbricoides* (43.3%) was recorded followed by hookworms (13.1%), *E. histolytica/dispar* (11.6%), *Giardia* sp. (10.8%), *T. trichura* (9.5%), *Cryptosporidium* spp. (3.1%), *H. nana* (1.8%), and *E. vermicularis* (0.5%)
(58)	Che Hasan et al.	2020	Carpal tunnel syndrome	Physical	WRMSD	Higher education	Office worker	Administration and secretarial occupations	O	2	1	Probable carpal tunnel syndrome (CTS) was 16.5% (*n* = 10)
(59)	Azmir and Yahya	2017	Hand arm vibration syndrome	Physical	WRMSD	Road	Hand-held grass-cutting worker	Elementary occupations	E	1	1	HAVS is diagnosed in Malaysia especially in agriculture sector
(60)	Ali et al.	2018	Hand arm vibration syndrome	Physical	WRMSD	Road	Hand-held grass-cutting worker	Elementary occupations	E	1	1	Daily vibration value depicted an exceeded exposure action value of 2.5 m/s^2^ for both hands and 80% of the workers experienced colour change in any of their fingers
(61)	Qamruddin et al.	2019	Hand arm vibration syndrome	Physical	WRMSD	Tyre shop	Tyre shop	Craft and related trade workers	G	1	1	Prevalence of the vascular, neurological, and musculoskeletal symptoms was 12.5% (95% CI 10.16 to 14.84), 37.0% (95% CI 30.31 to 43.69), and 44.5% (95% CI 37.61 to 51.38), respectively
(62)	Zamri et al.	2017	Low back pain	Physical	WRMSD	School	Teacher	Professionals	P	1	1	LBP and NSP among teachers in the past 12 months were 48.0% (95% (CI) 45.2%, 50.9%) and 60.1% (95% CI 57.4%, 62.9%)
(63)	Awang Lukman et al.	2019	Low back pain	Physical	WRMSD	NS	Commercial vehicle driver	Craft and related trade workers	H	2	1	Prevalence of LBP was 66.4%. The percentage of drivers who had frequent manual handling of heavy loads was 45.5% and those who handled heavy loads in awkward postures accounted for 86.4%.
(64)	Zamri et al.	2020	Low back pain	Physical	WRMSD	School	Teacher	Professionals	P	1	3	Prevalence of LBP at baseline and 12-month follow-up was 48.1% (95% CI: 45.6%, 51.7%) and 44.4% (95% CI: 40.6%, 48.0%), respectively
(65)	Ibrahim et al.	2019	Low back pain	Physical	WRMSD	Hospital	Healthcare worker	Associate professionals and technical officers	Q	1	1	989 (76.5%) nurses suffered from LBP
(66)	Tuan Lonik et al.	2017	Low back pain	Physical	WRMSD	Hospital	Healthcare worker	Personal service occupations	Q	1	1	Lifetime prevalence of LBP among the respondents was 65.0% (95% CI 57.1–72.9), with 12-month and 7-day prevalence rate of 88.8% (95% CI 83.6–94.0) and 20.3% (95% CI 13.6–26.9), respectively
(67)	Khan et al.	2020	Musculoskeletal	Physical	WRMSD	Higher education	University staff	NS	P	1	1	55.8% respondents (*n* = 234) reported neck pain (NP), (*n* = 196) 46.8% reported shoulder pain (SP), and (*n* = 308) 73.5% reported low back pain (LBP), respectively
(68)	Maakip et al.	2016	MSD	Physical	WRMSD	Office	Office worker	Administration and secretarial occupations	O	1	1	6-month period prevalence of MSD discomfort was 92.8% (95% CI: 90.2–95.2%)
(69)	Raghavendra Kamath et al.	2020	Musculoskeletal	Physical	WRMSD	Higher education	University staff	Associate professional and technical officers	C	2	1	Working on cutting machines and lathe in the machine shop and working in the foundry section record a RULA and REBA score of greater than 6, which states that there is a requirement of immediate action concerning the working posture on this equipment
(70)	Mohd Din et al.	2016	MSD	Physical	WRMSD	Forest	Army recruit	Armed forces	O	1	3	12% of the recruits were diagnosed with incident MSI and 80% reported incident MSD
(71)	Aziz et al.	2017	Musculoskeletal	Physical	WRMSD	Factory	Factory worker	Plant and machine operators and assemblers	C	NM	1	MSD prevalence for lower back (75.4%), upper back (63.2%), right shoulder (61.4%), and right wrist (60%)
(72)	Taib et al.	2017	Musculoskeletal	Physical	WRMSD	Clinic	Healthcare worker	Professionals	Q	2	1	The shoulders were most often affected by symptoms of MSDs (92.7%). MSDs of the neck and upper back were most likely to prevent these practitioners from engaging in normal activities (32.9%).
(73)	Amin et al.	2018	MSD	Physical	WRMSD	Hospital	Healthcare worker	Associate professionals and technical officers	Q	1	1	73.1% of the nursing staff experienced WRMSDs in at least one anatomical site 12 months prior to the study. 75% of nurses expressed emotional distress.
(74)	Labao et al.	2018	Musculoskeletal	Physical	WRMSD	NS	General worker	Elementary occupations	NS	2	1	Filipino migrant workers mostly complain of pain in the low back area (60%) and shoulder pain (60%), followed by pain in the upper back (48.3%) and neck pain (45%) in the last 12 months
(75)	Anwar et al.	2019	Musculoskeletal	Physical	WRMSD	Factory	Welder	Craft and related trade workers	C	2	1	25.9% had encountered neck pain, 11.1% experienced discomfort while performing repetitive actions, and 48.5% experienced discomfort and pain for both elbow/hand and wrist when lifting objects heavier than 5 kg
(76)	Alias et al.	2020	MSD	Physical	WRMSD	School	Teacher	Professionals	P	1	1	Prevalence for any parts of the body was 40.1%. The most affected part of the body was feet, with 32.5% for the past 12 months and 36.8% for the past 7 days.
(77)	Masri et al.	2017	MSD	Physical	WRMSD	Tea plantation	Tea plucker	Skilled agricultural, forestry, livestock, and fishery workers	A	1	1	Ergonomic risk factors faced by the tea puckers while performing their daily work tasks in the tea plantations are lifting, lifting with one shoulder, lifting above the shoulder, pushing, and pulling loads more than 25 kg
(78)	Shariat et al.	2018	Musculoskeletal	Physical	WRMSD	Office	Office worker	Administration and secretarial occupations	O	1	1	Significant association between pain severity in gender and right (*p*=0.046) and left (*p*=0.041) sides of the shoulders. There was also a significant association between BMI and severity of pain in the lower back area (*p*=0.047). It was revealed that total pain score in the shoulders was significantly associated with age (*p*=0.041).
(79)	Taib et al.	2018	Musculoskeletal	Physical	WRMSD	Hospital	Healthcare worker	Professionals	Q	2	1	32.6% of them reported that they have musculoskeletal discomfort at a single body region during the last year, 16.3% reported two regions, and 9.3% reported three regions where the most prevalent region affected was the neck area where 27.9% of the respondent reported they experienced symptoms or pain in this region, followed by wrists/hands (26.7%), lower back (19.8%), and upper back (14.0%)
(80)	Yahya and Zahid	2018	Musculoskeletal	Physical	WRMSD	Factory	Factory worker	Plant and machine operators and assemblers	C	2	1	30 respondents out of 36 respondents suffered from WMDs especially at shoulder, wrists, and lower back
(81)	Ng et al.	2019	Musculoskeletal	Physical	WRMSD	School	Teacher	Professionals	P	1	1	MSD during the previous 6 months was 80.1% (95% CI: 75.8–84.2%), with 80.5% of female and 77.5% of male teachers reporting symptomatic pain
(82)	Rahman et al.	2020	Musculoskeletal	Physical	WRMSD	Hospital	Healthcare worker	Associate professionals and technical officers	Q	2	1	Most of the respondents had been troubled with ache, pain, and discomfort at the neck, 54.9% (95% confidence interval 44.0%, 66.0%). In addition, they were troubled mainly with distress at the low back (34.1%) and the ankle or feet (34.1%) which had prevented the respondents from doing their regular job over the past 12 months.
(83)	Syed Abudaheer et al.	2020	Musculoskeletal	Physical	WRMSD	Higher education	University staff	Professionals	P	2	1	(*n* = 62) 73.8%. Shoulder, neck, and lower back region with slight variance in ranking. Shoulder is the highest at any time during the last 12 months. Neck has the highest prevalence at any time during the last seven days
(84)	Lim et al.	2021	Musculoskeletal	Physical	WRMSD	Municipal	Landscape workers	Elementary occupations	E	2	1	Overall prevalence of WRMSDs among landscape workers was 85.5%. The highest prevalence involving the shoulder (65.5%), followed by neck (23.6%), wrist/hand (23.6%), and lower back (20.0%) regions based on their self-reported WRMSD symptoms over the past 12 months
(85)	Yusof and Shahida	2021	Musculoskeletal	Physical	WRMSD	Factory	Factory worker	Craft and related trade workers	C	2	3	Workers experienced the highest discomfort in three body parts: (1) lower back, (2) shoulders, and (3) upper back. The discomfort felt by the workers was 74.36%, 8.96%, and 5.52% in the lower back, shoulders, and upper back, respectively.
(86)	Abdullahi et al.	2016	Sharp injury	Physical	Injury	Abattoir	Animal slaughter	Skilled agricultural, forestry, livestock, and fishery workers	A	2	1	Mean (SD) for occupational hazards = 2.32 (2.721). Proportion of injury by sharp equipment (20.0%), noise exposure (17.0%), and due to offensive odour within the abattoir premises (12.0%)
(87)	Hamid et al.	2016	Injury	Physical	Injury	Sport centre	Athlete	Professionals	R	1	1	83 injuries and 64 illnesses. Muscle strains and tears were the most common injuries followed by ligamentous injury and soft tissue contusion.
(88)	Ruslan et al.	2017	Injury	Physical	Injury	Palm oil plantation	Palm oil plantation worker	Plant and machine operators and assemblers	A	2	1	Prevalence of injury among palm oil mill workers was 39.4% with sprain and burn being the common types of injury reported. Press plant workers reported to have high cases of injuries. Majority of workers (78.8%) stated noise was the main hazard in the palm oil mill, followed by heat hazard.
(89)	Ishak et al.	2019	Sharps injury	Biology	Injury	Hospital	Healthcare worker	NS	Q	1	1	Works in the logging site and charcoal kiln could be carried out continuously with 25% of working efficiency on achieving maximum productivity and 75% of the rest needed, work in the nursery site it could be carried out continuously with 75% of working on achieving productivity and 25% of the rest needed
(90)	Achuthan et al.	2020	Heat stress	Physical	Injury	Forest	Forestry worker	Skilled agricultural, forestry, livestock, and fishery workers	A	NM	1	Works in the logging site and charcoal kiln could be carried out continuously with 25% of working efficiency on achieving maximum productivity and 75% of the rest needed, work in the nursery site it could be carried out continuously with 75% of working on achieving productivity and 25% of the rest needed
(91)	How et al.	2020	Heat stress	Physical	Injury	Farm	Farmer	Skilled agricultural, forestry, livestock, and fishery workers	A	2	1	Significant difference between HSI, blood pressure, and blood glucose levels among organic and conventional farmers. Both groups of farmers also have a significant association between blood glucose and blood pressure. Pesticide use can act as a synergistic effect, resulting in more significant health effects for those who were exposed to heat in their work environment.
(92)	Abidin et al.	2021	Sharp injury	Physical	Injury	Factory	Factory worker	Plant and machine operators and assemblers	C	1	1	Prevalence of occupational injury for the past 12 months was at 18%. The most often injured body parts were hands and legs while among the most common injury types were open wound, burns, and bleeding.
(93)	Ahmad et al.	2021	Occupational blood and body fluid exposure	Biology	Injury	Hospital	Healthcare worker	NS	Q	1	1	Prevalence of OBBE was 25.1% (95% confidence interval: 20.6–30.2), mostly due to percutaneous injuries, which were not reported to authorities
(94)	Lee et al.	2021	Injury	Physical	Injury	Sport centre	Athlete	Professionals	R	2	1	Pain was the predominantly observed symptom, with a predilection for the wrist, ring and middle fingers, and thumb. De Quervain's tenosynovitis was found in 53.8% (*n* = 21) of the subjects, with 52.4% and 42.9% of them experiencing pain during and after training, respectively.
(95)	Nawi et al.	2016	Injury	Physical	Injury	Palm oil plantation	Palm oil plantation worker	Elementary occupations	A	2	1	Using of manual tools should be avoided and plantation workers should be provided with ergonomic machines that can help them reduce their workload and injuries
(96)	Zerguine et al.	2018	Injury	Physical	Injury	Site	Construction workers	Elementary occupations	F	1	1	Work-related injuries in a one-year period was 22.6%, where most of the injuries were of moderate severity (39.7%) and falls from heights represented the main source (31.5%)
(97)	Mansor et al.	2019	Heat stress	Physical	Injury	Municipal	General worker	Elementary occupations	E	1	1	Percentage of respondents who experienced moderate to severe HRI was 44.1%
(98)	Sulaiman et al.	2019	Post-pesticide exposure	Chemical	Injury	Palm oil plantation	Palm oil plantation worker	Plant and machine operators and assemblers	A	1	1	Aware of the health hazards of pesticide use and suffered from symptoms (with mean duration of three days) such as vomiting, diarrhoea, skin irritation, and dizziness. Most of the workers responded that they did not receive any training in pesticide handling and used partial personal protective equipment (glasses, hats, shirt, and gloves) during working hours. Interestingly, a large percentage responded that they would not read the safety material even if it was provided.
(99)	Wahab et al.	2019	Sharps injury	Physical	Injury	Hospital	Healthcare worker	NS	Q	1	1	165 reported cases from 2013–2015. 65 (39.4%) were males, while 100 (60.6%) were females. The mean age was 27.41 (SD: 6.06). More than half of the reported sharps injury occurred among doctor, 113 (68.5%) specifically house officer; 89 (53.9%) followed by paramedic, 26 (15.8%) and others, 26 (15.8%). Mostly occurred in ward, 114 (69.1%)
(100)	Hamzah et al.	2016	Metal dust	Chemical	Respiratory	Factory	Factory worker	Plant and machine operators and assemblers	C	1	1	Only few workers (36.4%) were found to wear their masks all times during the working hours. There was an exposure-response relationship of cumulative metal dust exposure with the deterioration of lung function values
(101)	Hamsan et al.	2017	Pesticide concentrations	Chemical	Respiratory	Farm	Farmer	Skilled agricultural, forestry, livestock, and fishery workers	A	2	1	Hazard quotient (HQ) was less than 1 and the hazard index (HI) value was 3.86 × 10^−3^, indicating that the risk of pesticides related diseases was not significant. The lifetime cancer risk (LCR) for pymetrozine was at an acceptable level (LCR b 10^−6^) with 4.10 × 10^−8^.
(102)	Bakri et al.	2018	Respiratory illness	Chemical	Respiratory	Factory	Welder	Plant and machine operators and assemblers	C	2	1	Lung function decrement was established in linear regression for FEV1 and FEV1/FVC, respectively, although not statistically significant. Analysis conducted revealed the presence of the following trace elements concentration in ascending sequence: As < Al < Cu < Mn < Cr < Ni < Co < Fe (in the toenail) and Co < Al < Cu < Ni < As < Cr < Fe < Mn (in the cassette), respectively
(103)	Fandi et al.	2018	Air pollutants	Chemical	Respiratory	Road	Policemen	Personal service occupations	O	2	2	Mean personal exposure level of PM10 among the traffic policemen was 150.14 ± 130.66 *μ*g/m^3^ compared to only 84.14 ± 94.11 *μ*g/m^3^ in the comparative group. A median concentration of benzene documented significantly higher at the selected sampling roadsides areas (median = 0.157 ppm) than indoor office areas (median = 0.071 ppm).
(104)	Chean et al.	2019	Respiratory illness	Chemical	Respiratory	Road	Firefighters, traffic police	Personal service occupations	O	1	2	We recruited 706 participants—211 firefighters, 198 traffic police, and 297 from general population. Smokers had significantly higher scores than non-smokers in all SGRQ domains. Regardless of smoking status, the “occupationally exposed group” had higher symptoms score than the “occupationally unexposed group.”
(105)	Lim et al.	2019	Air pollutants	Chemical	Respiratory	Office	Office worker	Administration and secretarial occupations	O	1	1	9.6% of the workers had doctor-diagnosed asthma, 15.5% had wheezing, 18.4% had daytime attacks of breathlessness, and 25.8% had elevated FeNO (25 ppb). Median levels in office dust were 11.3 EU/mg endotoxin and 62.9 ng/g [1, 3]-b-glucan. After adjusting for personal and home environment factors, endotoxin concentration in dust was associated with wheezing (*p*=0.02) and rhinoconjunctivitis (*p*=0.007). The amount of surface dust (*p*=0.04) and [1, 3]-b-glucan concentration dust (*p*=0.03) was associated with elevated FeNO.
(106)	Bakar et al.	2020	Dust	Chemical	Respiratory	Hospital	Healthcare worker	NS	Q	2	1	Total dust concentration in the casting room is 3.402 ± 0.003 mg/m³ from area sampling and that for the personal air sampling is 5.573 ± 0.040 mg/m³ which are below 15 mg/m³ PEL.
(107)	Jamil et al.	2020	Air pollutants	Chemical	Respiratory	Road	Policemen	Personal service occupations	O	2	1	Occupational factors play a crucial role, and hence the authorities should take action in generating flexible working hours and the duration of services accordingly
(108)	Ratnasingam et al.	2016	Dust	Chemical	Respiratory	Factory	Factory worker	Plant and machine operators and assemblers	C	1	1	Highest dust emission from the sanding operation resulted in respiratory ailments among workers. The occurrence of injuries particularly to the hand, wrist, fingers, and forearm was due to the prevailing working conditions, safety climate, and workers' characteristics. The dust exposure levels and working conditions were much more severe in the bamboo furniture manufacturing industry.
(109)	Zakaria et al.	2019	Dust	Chemical	Respiratory	Factory	Factory worker	NS	C	2	1	Most of workers in the same environment are suffering from restrictive pattern of pulmonary disease.
(110)	Md Shakri et al.	2020	Endotoxin	Chemical	Respiratory	Factory	Factory worker	Plant and machine operators and assemblers	C	2	2	Mean concentration of endotoxin for areas was 0.26 (standard deviation (SD) = 0.12) EU/m^3^, whereas the mean personal inhalable endotoxin level among the rice millers was 0.29 (SD = 0.15) EU/m^3^. Post-shift lung function tests for FEV1/FVC measured appeared lower among rice millers (54%) compared to non-exposed workers (62%), but not statistically significant (*p*=0.313).
(111)	Salvaraji et al.	2020	Respiratory illness	Chemical	Respiratory	Municipal	Domestic waste collector	Elementary occupations	E	1	1	Respiratory symptoms were seen in 21% of the workers. The identified significant risk factors were determined as underlying chronic diseases (OR = 2.34; 95% CI = 1.054, 5.219) and contact with pets (OR = 1.87; 95% CI = 1.004, 3.288)
(112)	Hasan et al.	2016	Cardiovascular disease risk	Other	Cardiovascular disease	Office	Office worker	Administration and secretarial occupations	O	2	1	Respiratory symptoms were seen in 21% of the workers. The identified significant risk factors were determined as underlying chronic diseases (OR = 2.34; 95% CI = 1.054, 5.219) and contact with pets (OR = 1.87; 95% CI = 1.004, 3.288)
(113)	Lee et al.	2017	Cardiovascular disease risk	Other	Cardiovascular disease	School	Teacher	Professionals	P	1	1	MONO was 17.7% (95% confidence interval (CI), 15.3*e*20.4). Prevalence of metabolic syndrome among the normal weight and overweight participants was 8.3% (95% CI, 5.8*e*11.8) and 29.9% (95% CI, 26.3*e*33.7)
(114)	Kit et al.	2020	Overweight and obesity	Other	Cardiovascular disease	Clinic	Healthcare worker	NS	Q	1	1	49.9% of the healthcare workers were overweight or obese, 51.0% were at risk of having abdominal obesity, and 79.6% had a high body fat percentage
(115)	Kuan et al.	2020	Cardiovascular disease risk	Other	Cardiovascular disease	Hospital	Healthcare worker	NS	Q	1	1	47.4% of the subjects were of normal weight, 30.2% were overweight, 17.2% were obese and 5.2% were underweight
(116)	Rahimi et al.	2016	Cardiovascular disease risk	Other	Cardiovascular disease	Office	Rescue firefighter personnel	Personal service occupations	O	1	1	41.5% were normal, 44.8% were overweight, and 13% were obese. The percentage of 34.8% firefighters with WC values of more than 90 cm means that they were at greater risk to have cardiovascular and diabetes disease.
(117)	Samsuddin et al.	2016	Pesticide exposure	Chemical	Cardiovascular disease	Site	Healthcare worker	Personal service occupations	Q	1	2	Diazoxonase was significantly lower and ox-LDL was higher among pesticide-exposed workers than the comparison group. Age, body mass index (BMI), smoking, and pesticide exposure were independent predictors of brachial and aortic DBP and SBP. Pesticide exposure was also associated with heart rate, but not with PWV. Lipid profiles, PON1 enzymes, and ox-LDL showed no association with any of the CVS parameters.
(118)	Jeffree et al.	2016	Noise exposure	Physical	Hearing loss	Factory	Factory worker	Plant and machine operators and assemblers	C	2	2	Hearing impairment was significantly (*p* < 0.05) associated with older age, lower education level, high smoking dose, high occupational daily noise dose, longer duration of service, infrequent used of hearing protection device (HPD), and low perception of sound on HPD usage
(119)	Sam et al.	2017	Noise exposure	Physical	Hearing loss	Factory	Factory worker	Plant and machine operators and assemblers	C	2	1	Prevalence of HL was 73.3% and the prevalence of hearing impairment was 23.3%. Male workers (63.0%) had higher prevalence of HL than female workers (36.4%). Mean hearing threshold levels of HL respondents were significantly higher than respondents with normal hearing.
(120)	Selamat and Zulkifli	2016	Noise exposure	Physical	Hearing loss	Factory	Factory worker	Plant and machine operators and assemblers	C	2	1	Nearly all the identified work areas exceeded the action level of 85 dB (A) and four of these areas noise levels are more than 90 dB (A) which is the permissible exposure limit. For the questionnaire, it was found that annoyance topped the noise effect list with 51.4%, followed by stress with 40.0%, hearing deterioration (14.3%), and job performance deterioration (2.9%).

NS: not specified. SS = sample size, 1 = 150 and above, 2 =< 150, SD = study design, 1 = cross-sectional, 2 = case-control, 3 = others, Malaysia Standard Industrial Classification (MSIC) 2008, A: agriculture, forestry, and fishing, C: manufacturing, E: water supply; sewerage, waste management, and remediation activities, F: construction, G: wholesale and retail trade; repair of motor vehicles and motorcycle, H: transportation and storage, I: accommodation and food service activities, O: public administration and defense; compulsory social security, P: education, Q: human health and social work activities, and R: arts, entertainment, and recreation.

## Data Availability

The data that support the findings of this study are included within the article.
